RETRACTED

# Effects of the TLR4 signaling pathway on apoptosis of neuronal cells in diabetes mellitus complicated with cerebral infarction in a rat model

**DOI:** 10.1038/srep43834

**Published:** 2017-03-08

**Authors:** Chao Li, Li-He Che, Tie-Feng Ji, Lei Shi, Jin-Lu Yu

**Affiliations:** 1 Department of Neurology, The First Hospital of Jilin University, Changchun 130021, P.R. China; 2 Department of Infectious Diseases, The First Hospital of Jilin University, Changchun 130021, P.R. China; 3 Department of Radiology, The First Hospital of Jilin University, Changchun 130021, P.R. China; 4 Department of Neurosurgery, The First Hospital of Jilin University, Changchun 130021, P.R. China

## Abstract

This study aims to explore the effects of the TLR4 signaling pathway on the apoptosis of neuronal cells in rats with diabetes mellitus complicated with cerebral infarction (DMCI). A DMCI model was established with 40 Sprague Dawley rats, which were assigned into blank, sham, DM + middle cerebral artery occlusion (MCAO) and DM + MCAO + TAK242 groups. Superoxide dismutase (SOD) activity and malondialdehyde (MDA) content were measured. A TUNEL assay was applied for detecting cell apoptosis, and Western blotting was used for detecting the expression of TLR4, TNF-α, IL-1β and apoptosis-related proteins. Compared with the blank and sham groups, there was an increase in cell apoptosis, expression of Bcl-2, Bax, cleaved caspase-3, TNF-α, IL-1β and TLR4 proteins and MDA content and a decrease in SOD activity in the DM + MCAO and DM + MCAO + TAK242 groups. Compared with those in the DM + MCAO group, rats in the DM + MCAO + TAK242 group exhibited an increase in SOD activity and a decrease in cell apoptosis, expression of Bcl-2, Bax, cleaved caspase-3, TNF-α, IL-1β and TLR4 proteins and MDA content. Inhibition of the TLR4 signaling pathway reduces neuronal cell apoptosis and nerve injury to protect the brain.

As a cause of diabetic angiopathy, diabetes mellitus (DM) is an independent risk factor for cerebral infarction^1^. For example, in one study, DM patients were shown to have a 1.5 to 3-times higher risk of stroke, especially cerebral infarction, than non-diabetic subjects^2^. In addition, cerebral infarction is one of the common complications of diabetes; approximately 15 cases of cerebral infarction in 2000 diabetes patients occurred annually, and the incidence is rising significantly^3^. Furthermore, DM is often complicated with acute cerebral infarction (DMCI), and the recurrence rate, morbidity and mortality of DMCI are high, with poor prognosis^1^. Clinically, the neurological deficit in DMCI patients is characterized by a predominance of a motor deficit, mainly including weakness, numbness, limitation of one side limb, motion, dyslalia and alalia^4^. With respect to the pathogenesis of DMCI, the long-term high blood glucose concentration is general believed to lead to vascular wall damages, an increase in blood viscosity and vascular sclerosis, which all eventually lead to a vascular infarction^5^,^6^. Currently, the molecular mechanism of DMCI still ambiguous, and several studies have reported that it may be associated with vascular cell adhesion molecule-1 (VCAM-1) and inflammatory factors^7^,^8^. The immune inflammatory response is consistently involved throughout diabetic vascular disease, especially Toll-like receptor 4 (TLR4)^9^.

RETRACTED

Apart from special recognition of biological and non-biological stimuli, TLR4 is not only able to induce and amplify the inflammatory response but also plays a vital role in cell proliferation, differentiation and apoptosis^10^. Previous studies have demonstrated that TLR4 could mediate the inflammatory response of cerebral ischemia via activating the nuclear factor-κB (NF-κB) pathway and downstream inflammatory factors to aggravate ischemic brain damage, which results in cerebral stroke^11^,^12^. In addition, TLR4 can be involved in hyperinsulinemia, insulin resistance, lipid metabolism disorder, endothelial cell dysfunction and blood coagulation, which all affect diabetic vascular disease^13^,^14^. However, there has been no research on the effects of the TLR4 signaling pathway on DMCI. Therefore, this study aims to explore the effects of the TLR4 signaling pathway on apoptosis of neuronal cells via introducing TAK242 (a TLR4 signaling inhibitor) and establishing a DMCI rat model to provide a theoretical basis for the pathological mechanism for DMCI and the development of a targeted drug treatment.

## Materials and Methods

### Ethics statement

Animal experiments were conducted in strict accordance with the approved animal protocols and guidelines established by the Medicine Ethics Review Committee for animal experiments of The First Hospital of Jilin University. All efforts were made to minimize the suffering of animals.

### Subjects

A total of 40 male Sprague Dawley (SD) rats (4–6 weeks old, 200~250 g) were purchased from the SJA Lab Animal Limited Company (Changsha, Hunan, China). Rats were fed with pellet food, had free access to drinking water at 25–26 °C, and were maintained at a relative humidity of 60–70%. Clean padding was changed twice a week. All animals were kept in standard feeding rooms under the same condition of feed, water supply, light and temperature.

### Model establishment and grouping

SD rats were injected with alloxan (100 mg/kg) intraperitoneally for 2 days. The fasting blood glucose was measured using the glucose oxidase method at 72 h after the last administration. Rats with fasting blood glucose greater than 16.7 mmol/L were used as the DM model. After 5 weeks of a high-fat and high-sugar diet, the rats were injected with 20% urethane intraperitoneally and anaesthetized. The middle cerebral artery occlusion (MCAO) model was established using the suture method. At room temperature 24 ± 1 °C, rats under anesthesia were fixed on an operating table in a supine position. A cervical median incision was made. The common carotid artery (CCA), external carotid artery (ECA) and internal carotid artery (ICA) on the right side were isolated and exposed. The proximal end of the CCA and the root of the ECA were ligated. A syringe needle was used to pierce the distal end of the upper wall of the CCA to insert a 0.25-mm nylon suture via the ICA to the arterial origin until meeting resistance. The nylon suture was fixed, and the incision was sutured. After the rats awoke, those walking in a circle to the left and those that exhibited paralysis of the left limbs were considered to have had a successful MCAO and were used further in the experiment.

RETRACTED

A total of 40 SD rats were randomly assigned into the blank group, the sham group, the DM + MCAO group and the TLR4 inhibitor group (DM + MCAO + TAK242). Each group contained 10 rats. Rats in the blank group had no treatment. Rats in the DM + MCAO and DM + MCAO + TAK242 groups were used for the above operation. Rats in the sham group had the same operation with only a 10-mm insert depth for 1 min in which the suture was not fixed. Rats in the blank group were fed with a normal diet, while rats in the sham, DM + MCAO and DM + MCAO + TAK242 groups were fed with high-fat and high-sugar diets (containing 10% lard, 10% yolk powder and 20% sucrose). In the DM + MCAO + TAK242 group, rats were treated with an intraperitoneal injection of 3 mg/kg TAK242 (MedChemExpress Company, New Jersey, USA), which is a specific TLR4 inhibitor. The injection was conducted once a day for 5 days.

### Neurological severity score (NSS)

Behavior observation was performed when every rat was conscious 4 h after the operation. According to Zausinger *et al*.^15^, a higher score indicated a severer neurological injury. The scores were as follows: a score of 0 indicated that there was no neurological function impairment; 1 indicated that the rats showed contralateral forelimb flexion and adduction during tail suspension, that is, symptoms of slight neurological function impairment; 2 indicated that the rats were walking in a circle to the side of the cerebral injury in a head-to-rear shaped posture but were in a normal posture at rest, i.e., moderate symptoms of neurological function impairment; 3 indicated that the rats fell to the side of the cerebral injury, i.e., severe symptoms of neurological function impairment; and a score of 4 indicated that the rats had decreased levels of consciousness and displayed no spontaneous activity, i.e., very severe symptoms of neurological function impairment.

RETRACTED

### Brain tissue collection

Five days after modeling of MCAO, the rats were injected with 20% urethane intraperitoneally and anaesthetized. The left ventricle was perfused with normal saline (100 mL) to wash the blood vessel and then perfused with 1.5% glutaraldehyde (200 mL) and 4% paraformaldehyde (200 mL) for 1 h. The penumbra region was normalized using the equivalent location method among groups. Cortical tissue blocks were collected from the olfactory bulb point (7–13 nm) and 1/3 sagittal fissure to the lateral fissure of the right hemisphere at low temperature.

### Measurement of the cerebral infarction volume and cerebral water content

The brain tissue was frozen at −20 °C for 5 min. The frontal pole was cut off. Brain samples were sequentially sliced every 3 mm, then placed in 2% triphenyltetrazolium chloride (TTC) solution and incubated at 37 °C for 20 min. The stained brain slices were fixed using 4% paraformaldehyde for 10 h and photographed. A BI-2000 Medical image analysis system (Olympus Optical Co., Ltd, Tokyo, Japan) was used to calculate the volume of the cerebral infarction. The infarction volume of each brain slice was calculated by multiplying the infarct area of the ipsilateral cerebral infarction by its thickness. The total cerebral infarction volume was the sum of the infarction volume of each brain slice. The relative volume of the cerebral infarction = total cerebral infarction volume/volume of the contralateral brain tissue. The dry-wet method was performed to determine the cerebral water content. Fresh brain tissue was weighed to obtain the wet weight. Then, the fresh tissue was dried in an oven at 100 °C for 24 h and weighed again to obtain the dry weight. Cerebral water content (%) = (wet weight − dry weight)/wet weight × 100%.

### Nissl staining

Rat brain slices from each group were observed under a microscope (Olympus Optical Co., Ltd, Tokyo, Japan) to select the slice with the typical hippocampal formation, followed by sequentially slicing 3 sections at a thickness of 5 μm per section. After immersion in distilled water for 2 min, sections were placed in a humidified box in a water bath at 50 °C. Then, the Nissl staining solution (Hope Biotechnology Company, Qingdao, China) was centrifuged for 2 min. The slices were stained for 6 min with the addition of 10 μL of Nissl staining solution. After the slices were washed with distilled water 2 times, the slices were placed in graded ethyl alcohol (95%, 70%, and 70%, sequentially) for 5 s and sealed, followed by observation under a microscope. A total of 3 sections at the same level were selected from different samples, and 5 views were randomly selected from the portions to be counted in each slice to count the number of normal neurons in the hippocampal CA1 area for an average value. The density of the neurons in the hippocampal CA1 area = the number of normal neurons in the CA1 area/the total length of the CA1 area (mm).

RETRACTED

### Determination of superoxide dismutase (SOD) activity and malondialdehyde (MDA) content

The brains of rats were collected, dried and weighed before preparing a 10% homogenate by adding ice physiological saline at a volume of 1: 9 (w: v). The homogenate was centrifuged at 3000 rpm for 15 min at 4 °C. The supernatant was collected and stored at −80 °C for further testing. According to the kit instructions (Jianchen Biological Institute, Shanghai, China), the activity of SOD and the content of MDA were determined using spectrophotometry. SOD activity was detected using the xanthine oxidase method. In the brain homogenate samples, when the SOD inhibition rate of each milligram in a 1-mL reaction liquid was 50%, the corresponding content of SOD was determined to be a single activity unit of SOD (U/mg protein). The MDA content was determined using the thiobarbituric acid (TBA) method.

### Terminal deoxy-nucleotidyl transferase mediated dUTP-nick-end-labeling (TUNEL) assay

A TUNEL assay was conducted to detect apoptosis. The brain tissue samples were dewaxed to water and treated with freshly prepared 2% H_2_O_2_ at room temperature for 10 min. Then, the samples were treated with 20 μg/ml non-deoxyribonuclease (DNase) proteinase K (Merck Drugs & Biotechnology Inc., Darmstadt, Germany) for 30 min at 37 °C to remove the nuclease, followed by washing with PBS three times for 4 min each. Terminal deoxynucleotidyl transferase (TdT) (F. Hoffmann-La Roche & Co., California, USA) and biotin-dUTP (F. Hoffmann-La Roche & Co., California, USA) were added to the samples, and the mixtures were incubated in the dark at 37 °C for 60 min, followed by PBS washing. Labeling reaction termination solution was added to the samples, followed by incubation at 37 °C for 60 min and washing with PBS. Streptavidin-HRP enzyme (F. Hoffmann-La Roche & Co., California, USA) (10 μL) and Biotin-dUTP (490 μL) were mixed and added onto the sections, and the sections were incubated in the dark for 60 min at 37 °C. After PBS washing, the 3′-diaminobenzidine (DAB) solution (F. Hoffmann-La Roche & Co., California, USA) was used to develop the stain. The samples were counterstained with hematoxylin (Solarbio science & technology Co., Ltd., Beijing, China). The samples were washed with PBS, dehydrated, mounted in neutral resins and photographed.

RETRACTED

### Western blotting

Brains were weighed, and pre-cooled RIPA lysis buffer (1 mL/100 mg) was added. After the brains were homogenized, the homogenate was centrifuged at 12000 rpm for 10 min at 4 °C. The supernatant was diluted, and the protein expression was determined. The loading buffer was added to the tissue proteins to adjust the concentration and volume, and later, 20 μL of samples were collected for electrophoresis in a 12% polyacrylamide gel. After electrophoresis, the samples were transferred to membranes and blocked with T-TBS containing 5% bovine serum albumin (BSA) at room temperature. The blocking buffer was removed, and the membranes were placed into a plastic groove and incubated overnight with primary antibodies against Bcl-2, Bax, cleaved caspase-3, TNF-α, IL-1β, TLR4 and β-actin (Abcam Inc., Cambridge, UK) at 4 °C. The next day, the membranes were rinsed three times for 10 min with TBS-T. The same method was carried out to incubate the membranes with the second antibody in a shaker for 1 h, followed by washing three times with TBS-T for 15 min each. The chemoluminescence A solution and B solution were mixed in a 1: 1 ratio and added onto the nitrocellulose filter (NC) membrane. Finally, the developing substrate was added for film development. The relative optical density of the bands was analyzed using Image J software.

### Statistical analysis

The statistical analysis was performed using SPSS 21.0 (SPSS Inc., Chicago, IL, USA) software. Data were expressed as the mean ± standard deviation (SD). Comparison among groups was analyzed by one-way analysis of variance, and pairwise comparison by *t*-test. *P* < 0.05 was considered statistically significant.

## Results

### Evaluation of the DM model and MCAO model

The fasting blood glucose of rats (n = 30) in the sham, DM + MCAO and DM + MCAO + TAK242 groups was more than 16.7 mmol/L. No animals died in the following month, and the success rate was 100%. After the establishment of the DM model, the rats showed weight loss, an increase in water intake, food intake and urine volume as well as dirty fur and frequent fluctuations in high blood glucose. The MCAO model was established successfully in DM model rats. No animals died, and rats in the DM + MCAO and DM + MCAO + TAK242 groups (n = 20) displayed neurological deficits of different severities. The DMCI model was established with a success rate of 100%.

RETRACTED

### Blood glucose changes in rats of the four groups

The blood glucose changes in the rats of the four groups before and after intraperitoneal injection of alloxan are shown in Fig. 1. There was no difference between rats in the DM + MCAO and DM + MACO + TAK242 groups and rats in the blank and sham groups (all *P* > 0.05). One week after alloxan injection, the blood glucose of rats in the sham, DM + MCAO and DM + MACO + TAK242 groups was higher than that of the blank group (all *P* < 0.05). The blood glucose levels of the rats in the DM + MCAO and DM + MACO + TAK242 groups were not significantly different (*P* > 0.05).

### Neurological severity scores of rats among the four groups

In the blank and sham groups, no neurological deficits were found, and the corresponding neurological score was 0. In contrast, in the DM + MCAO and DM + MCAO + TAK242 groups, rats had different degrees of contralateral hemiplegia shown by ptosis, mydriasis, paralysis of the left forelimb, adduction flexion of the left forelimb upon tail suspension and falling to the paralyzed side when walking. Compared with the neurological scores of the blank and sham groups, those of the rats in the DM + MCAO and DM + MCAO + TAK242 groups were significantly higher (all *P* < 0.05). The neurological scores of rats in the DM + MCAO + TAK242 group were lower than that of the rats in the DM + MCAO group (*P* < 0.05) (Fig. 2).

### Cerebral infarction volume and cerebral water content in rats among the four groups

There was no infarct present in the blank and sham groups, but a pale infarct was found in the DM + MCAO and DM + MCAO + TAK242 groups (Fig. 3). Moreover, the infarct volume ratio was the highest in the DM + MCAO group, especially in cases of severe infarcts that covered almost half of the brain. Compared with those of the blank and sham groups, the infarction volume and cerebral water content was increased in the DM + MCAO and DM + MCAO + TAK242 groups (all *P* < 0.05). The infarction volume and cerebral water content were lower in the DM + MCAO + TAK242 group than in the DM + MCAO group (all *P* < 0.05), indicating that rats exhibited brain edema after cerebral infarction and that the TLR4 inhibitor reduced the infarct ratio.

### Neuronal damage in rats among the four groups

The neuronal damage observed by Nissl staining (Fig. 4) showed that, in the blank and sham groups, a large number of Nissl bodies (purple triangle) were arranged in order. In the DM + MCAO and DM + MCAO + TAK242 groups, the number of Nissl bodies was reduced, and the cells were no longer arranged in an orderly manner. The number of neurons was reduced, and the residual neurons exhibited indications of cell necrosis such as nuclear concentration, loose tissue, and light staining of the cytoplasm. Neurons around the infarct exhibited edema. The number of Nissl bodies in the DM + MCAO + TAK242 group was higher, and the cells were relatively more ordered with fewer cells exhibiting signs of necrosis than in the DM + MCAO group, indicating that the TLR4 inhibitor could protect and repair hippocampal neurons.

RETRACTED

### SOD activity and MDA content in the brain tissue among the four groups

The antioxidant enzyme SOD activity and MDA content in the brain tissue of the four groups are shown in Fig. 5. No significant differences were found between the blank and sham group. In the DM + MCAO and DM + MCAO + TAK242 groups, SOD activity in the brain tissue was greatly decreased, while MDA content was notably increased compared with that of the blank and sham groups (all *P* < 0.05). Compared with the SOD activity and MDA content in the DM + MCAO group, there was a great increase in SOD activity and an obvious decrease in MDA content in the DM + MCAO + TAK242 group (all *P* < 0.05), indicating that the inhibition of the TLR4 signaling pathway could significantly improve the antioxidant capacity of rats, thereby protecting the brain tissue.

### Apoptosis of rat brain neuronal cells among the four groups

In the blank and sham groups, TUNEL - positive apoptotic cells were distributed sporadically, while in the DM + MCAO and DM + MCAO + TAK242 groups, the number of positive apoptotic cells was greatly increased, mainly in neuronal cells around the cerebral infarction (Fig. 6). The number of apoptotic neuronal cells was higher in the DM + MCAO and DM + MCAO + TAK242 groups than in the blank and sham groups (all *P* < 0.05). Compared with the number of apoptotic neurons in the DM + MCAO group, the number of apoptotic neuronal cells was reduced in the DM + MCAO + TAK242 group (*P* < 0.05), suggesting that the TLR4 inhibitor can reduce the apoptosis of neuronal cells.

### The expression of apoptosis-related proteins and TLR4 signal-related proteins in the rat brain among the four groups

There were no significant differences in the protein expression between the blank and sham groups (*P* > 0.05). In contrast, in the DM + MCAO and DM + MCAO + TAK242 groups, there was an evident increase in the expression of apoptosis-related proteins (Bcl-2, Bax and cleaved caspase-3) and proteins downstream of the TLR4 signal (TNF-α and IL-1β) as well as TLR4 protein in the rat brain tissue samples compared with that of the blank and sham groups (all *P* < 0.05). Compared with the expression in the DM + MCAO group, the expression of Bcl-2, Bax, cleaved caspase-3, TNF-α, IL-1β and TLR4 proteins was greatly reduced in the DM + MCAO + TAK242 group (all *P* < 0.05) (Fig. 7).

RETRACTED

## Discussion

TLR4, which transmits an inflammatory signal, functions as a portal protein involved in diabetic angiopathies via mediating a signaling pathway that activates the transcription and synthesis of inflammatory factors and has become a new attractive field for studying DM and related complications^13^,^14^. However, it is still unknown how TLR4 affects DMCI. Therefore, this study evaluated the effects of TLR4 on DMCI in terms of blood glucose, neurological function, antioxidant ability, cerebral infarct volume ratio, inflammatory factors, neuronal apoptosis and relative protein expression.

In this study, we established a DMCI rat model and found that, compared with that of the DM + MCAO group, the blood glucose of rats in the DM + MCAO + TAK242 group was slightly decreased but not significantly different, indicating that the TLR4 inhibitor cannot reduce the blood glucose of DMCI rats. In addition, Singh, Boden and Rao reported that high glucose increased the expression of TLR-4^16^. Moreover, other studies confirmed that high glucose could trigger the TLR4 signaling pathway to activate a related receptor^17^,^18^. All of these studies showed that blood glucose is upstream of TLR4, and that the TLR4 inhibitor alone cannot change blood glucose content.

In addition, this study found that in the DM + MCAO + TAK242 group, SOD activity was higher, while MDA content was lower than that in the DM + MCAO group. MDA can reflect the reactive oxygen level *in vivo*, which indirectly shows the severity of the oxidative stress injury, while SOD functions as an antioxidant enzyme to protect cells from oxidative stress damage^19^. Our results elucidated that inhibition of the TLR4 signaling pathway improves the antioxidant capacity of rats. The inhibition of the TLR4 signaling pathway may result in a decrease in lipopolysaccharide-induced reactive oxygen species production, which is mediated by TLR4, to reduce the oxygen radical damage to the body, thereby playing a protective role in the brain tissue^20^.

In addition, this study reported that the inhibition of the TLR4 signaling pathway can reduce neural function damage and the apoptosis of neurons, which may be related to the involvement of the TLR4 signaling pathway in regulating apoptosis-related proteins and the expression of TLR4 downstream proteins. Molecularly, the inhibition of the TLR4 signaling pathway leads to a significant decline in the expression levels of apoptosis-related proteins such as Bcl-2, Bax and cleaved caspase-3 in the rat brain. Bcl-2 and Bax, belonging to pro- or anti-apoptotic gene families, mediate apoptosis mainly via regulating the release of cytochrome C and the mitochondrial pathway, as well as by mediating caspases^21^,^22^, a type of cysteine-containing aspartate-specific protease, in which caspase-3, as the executor of apoptosis, is a key protease in mammalian cell apoptosis^23^. The TLR4 signaling pathway exerts effects on the expression of apoptosis-related proteins Bax and Bcl-2 to initiate apoptosis via activating the transcription of inflammatory factors downstream of TLR4^24^. Currently, there are two explanations for the mechanism of the involvement of TLR4 in neuronal apoptosis: TLR4 can participate in neuronal apoptosis through the Akt/FoxO3a/Bim signaling pathway^25^; TLR4 can mediate caspase-3 to be involved in nerve injury and neuronal apoptosis^20^. In addition, the expression of downstream inflammatory factors TNF-α and IL-1β evidently decreased along with the decrease in the expression of TLR4, which may be related to the molecular mechanism of TLR4, that is, LPS-induced TLR4 leads to the secretion of cytokines such as IL-1β and TNF-α^26^.

RETRACTED

In summary, inhibition of the TLR4 inflammatory signaling pathway can reduce the expression of apoptosis-related proteins in brain tissue, neuronal apoptosis and nerve injury in DMCI rats to protect the brain. Therefore, the development of targeted drugs that inhibit the TLR4 signaling pathway is expected to treat and prevent DMCI.

## Additional Information

**How to cite this article:** Li, C. *et al*. Effects of the TLR4 signaling pathway on apoptosis of neuronal cells in diabetes mellitus complicated with cerebral infarction in a rat model. *Sci. Rep.* **7**, 43834; doi: 10.1038/srep43834 (2017).

**Publisher's note:** Springer Nature remains neutral with regard to jurisdictional claims in published maps and institutional affiliations.

## Figures and Tables

**Figure 1:** The blood glucose changes of rats in the four groups. *Compared with the blank group, *P* < 0.05.

**Figure 2:** The neurological scores of rats in the four groups. *Compared with the blank group, *P* < 0.05; ^#^compared with the sham group, *P* < 0.05; ^&^compared with the DM + MCAO group, *P* < 0.05; DM, diabetes mellitus; MACO, middle cerebral artery occlusion.

**Figure 3:** The TTC staining of brain tissue (**A**), cerebral infarction volume (**B**) and cerebral water content (**C**) of rats in the four groups. *Compared with the blank group, *P* < 0.05; ^#^compared with the sham group, *P* < 0.05; ^&^compared with the DM + MCAO group, *P* < 0.05; TTC, triphenyltetrazolium chloride; DM, diabetes mellitus; MACO, middle cerebral artery occlusion.

**Figure 4:** Nissl staining of hippocampal neurons in the CA1 area in the four groups (200×).

RETRACTED

**Figure 5:** The SOD activity (**A**) and MDA content (**B**) of rats in the four groups. *Compared with the blank group, *P* < 0.05; ^#^compared with the sham group, *P* < 0.05; ^&^compared with the DM + MCAO group, *P* < 0.05; SOD, superoxide dismutase; MDA, malondialdehyde; DM, diabetes mellitus; MACO, middle cerebral artery occlusion.

**Figure 6:** The cell apoptosis of brain neuronal cells of rats in the four groups by TUNEL staining (**A**) and the quantification of staining (**B**). *Compared with the blank group, *P* < 0.05; ^#^compared with the sham group, *P* < 0.05; ^&^compared with the DM + MCAO group, *P* < 0.05; TUNEL, terminal deoxy-nucleotidyl transferase mediated dUTP-nick-end-labeling; DM, diabetes mellitus; MACO, middle cerebral artery occlusion.

**Figure 7:** The protein expressions of apoptosis- and TLR4 signal-related proteins of the rat brains in the four groups by Western blotting (**A**) and the analysis histograms (**B**). *Compared with the blank group, *P* < 0.05; ^#^compared with the sham group, *P* < 0.05; ^&^compared with the DM + MCAO group, *P* < 0.05; TLR4, toll-like receptor 4; DM, diabetes mellitus; MACO, middle cerebral artery occlusion.
